# Unilateral Facial Paralysis With Facial Nerve Enhancement on MRI in a Patient With Guillain-Barré Syndrome: A Case Report

**DOI:** 10.7759/cureus.91042

**Published:** 2025-08-26

**Authors:** Aaron Creswell, Abigail Zaratan, Darius Shahbazi, Shahin Shahbazi

**Affiliations:** 1 Neurology, California Northstate University College of Medicine, Elk Grove, USA; 2 Clinical Medicine, California Northstate University College of Medicine, Elk Grove, USA; 3 Hospital Medicine, Kansas City University College of Osteopathic Medicine, Kansas City, USA; 4 Hospital Medicine, Kaiser Roseville Medical Center, Sacramento, USA

**Keywords:** autoimmune demyelination, bell's palsy, facial palsy, guillain-barré syndrome (gbs), post-infectious demyelination

## Abstract

Guillain-Barré syndrome (GBS) represents a spectrum of inflammatory polyradiculoneuropathies. Several variants have been reported with distinct symptom profiles. Cranial nerve involvement is relatively common, but it most often presents as bilateral facial nerve palsy at onset. We describe the case of a 66-year-old man who initially presented with extremity paresthesia that rapidly progressed to leg weakness and hyporeflexia. The diagnosis of GBS was confirmed by cerebrospinal fluid analysis, and he was treated with intravenous immunoglobulin. Following treatment, however, he developed facial hemiplegia, which was associated with facial nerve enhancement on MRI. This case represents one of the few reports of delayed-onset unilateral cranial nerve palsy in GBS, further distinguished by the rare finding of facial nerve enhancement on MRI. Awareness of such uncommon variants is important, as they may influence both morbidity and mortality.

## Introduction

Guillain-Barré syndrome (GBS) describes a heterogeneous group of post-infectious inflammatory disorders characterized by autoimmune demyelination of the peripheral nerves. A variety of infectious agents have been implicated, including more recently COVID-19 and its vaccines, but the most common triggers remain *Campylobacter jejuni*, influenza, cytomegalovirus, Epstein-Barr virus, and *Mycoplasma pneumoniae* [1]. The pathophysiology is multifactorial and not yet fully understood, though it likely involves molecular mimicry leading to immune-mediated myelin damage. Many cases are also associated with anti-ganglioside antibodies [1]. The classic presentation of GBS typically begins several weeks after a respiratory or diarrheal illness with symmetric, ascending paralysis. However, several variants with distinct symptom profiles have been described, including Miller-Fisher syndrome (ophthalmoplegia, ataxia, areflexia), the pharyngeal-cervical-brachial form, and acute motor axonal neuropathy, which involves only motor axons [2]. Cranial nerve involvement occurs in about 50% of patients with GBS, most often presenting as bilateral polyneuropathy, including early facial diplegia [3]. This case report adds to the very limited number of cases where unilateral facial weakness, closely resembling Bell’s palsy, developed weeks after the initial illness, and in this case, following completion of immunoglobulin therapy. Recognition of this rare complication is important for both clinicians and patients, as it may affect disease management, contribute to complications, and influence outcomes.

## Case presentation

This case report describes a 66-year-old man with a history of chronic back pain and mild alcohol use disorder who presented to the emergency department with bilateral numbness in his fingers and toes, beginning four days after starting azithromycin and albuterol for an upper respiratory tract infection. He also reported recent-onset left arm soreness and upper back pain. Physical examination was unremarkable except for tenderness to palpation in the mid-thoracic back, left of the midline. Laboratory studies, including complete blood count, metabolic panel, troponins, and urinalysis, were within normal limits, and the electrocardiogram (EKG) was unremarkable. He was discharged with a diagnosis of back pain and advised to discontinue azithromycin. 

Two days later, he returned to the emergency department with persistent tingling in the soles of his feet and toes, new-onset low back pain, progressive leg weakness, and difficulty walking, leading to two falls. On examination, head, neck, cardiovascular, pulmonary, and abdominal findings were normal. The musculoskeletal exam showed no spinal tenderness and a normal range of motion. Neurologically, the patient was alert and oriented, with decreased sensation on the plantar surfaces of both great toes. Motor strength was 4/5 in bilateral hip flexors and extensors, and 5/5 in the knees, ankles, and toes. Straight leg raise and resisted movements elicited pain. He was unable to ambulate steadily, and deep tendon reflexes were diminished (1+) at the Achilles and patellar tendons bilaterally. Laboratory studies again remained within normal limits. MRI of the lumbar spine (Figure 1) revealed multilevel degenerative changes with mild canal stenosis. Severe right-sided and moderate-to-severe left-sided neural foraminal narrowing was noted at L4-L5, with moderate narrowing bilaterally at L3-L4 and L5-S1.

**Figure 1:** MRI of the lumbar spine. (A) T2-weighted axial view showing right- and left-sided neural foraminal narrowing. (B) T2-weighted sagittal view showing multilevel degenerative changes (red) and mild canal stenosis (blue)

Neurology was consulted the following day after the patient’s symptoms progressed to include upper extremity numbness and worsening lower extremity weakness. On neurological examination, the patient was alert, with intact pinprick, temperature, and vibration sensation. Motor strength was 5/5 in the arms and hands but reduced to 4/5 in the lower extremities, with greater weakness on the left. Deep tendon reflexes were absent in the bilateral triceps, brachioradialis, patellar, and ankle regions, with a +1 response in the right biceps and an absent response in the left biceps. Based on the patient’s clinical presentation and progression, GBS was the leading differential diagnosis, and intravenous immunoglobulin (IVIG) at 400 mg/kg/day was initiated empirically for five days.

Further workup included a lumbar puncture, which demonstrated albuminocytologic dissociation, supporting the diagnosis of GBS (Table 1). Additional studies, including erythrocyte sedimentation rate (ESR), C-reactive protein (CRP), thyroid-stimulating hormone (TSH), vitamin B12, and folic acid, were performed to rule out other causes of neuropathy, all of which were within normal limits (Table 2). A cerebrospinal fluid (CSF) titer for West Nile virus was also unremarkable (Table 1).

**Table 1:** Cerebrospinal fluid (CSF) analysis

Parameter	Patient values	Reference range
Color	Colorless	Colorless
Appearance	Clear	Clear
RBC count	1/uL	0-5/uL
Total nucleated cells	1/uL	0-5/uL
CSF protein	152 mg/dL	15-45 mg/dL
CSF glucose	75 mg/dL	40-70 mg/dL
West Nile virus IGG	0.37 mg/dL	<1.3 mg/dL
West Nile virus IGM	0.03 mg/dL	<0.9 mg/dL

**Table 2:** Results of laboratory tests obtained for evaluation of neuropathy

Parameter	Patient values	Reference range
Erythrocyte sedimentation rate (ESR)	5 mm/h	0-15 mm/h
C-reactive protein (CRP)	0.3 mg/dL	<1 mg/dL
Thyroid-stimulating hormone (TSH)	0.8 mIU/L	0.4-4.0 mIU/L
Vitamin B1	173 nmol/L	74-222 nmol/L
Vitamin B12	508 pg/mL	110-1500 pg/mL
Folic acid	>15 ng/mL	>4 ng/mL

Management included monitoring respiratory muscle strength with forced vital capacity (FVC) and negative inspiratory force (NIF) measurements. During IVIG therapy, the patient developed lower extremity and back muscle pain, which was managed symptomatically. Over the five-day treatment course, he showed mild improvement in lower extremity strength and gradual recovery of upper extremity deep tendon reflexes. Two days after completing IVIG, the patient developed right-sided facial droop, ptosis, and nystagmus. Neurological examination revealed no altered mental status. Sensation to light touch and pinprick was decreased in the right upper extremity, though facial sensation and upper extremity strength were preserved. Mild dysarthria was noted without aphasia. Additional findings included excessive drooling and incomplete closure of the right eyelid. Given the concern for stroke versus cranial nerve involvement in GBS, an MRI of the head was obtained. Imaging (Figure 2) revealed a small 3 mm focus of enhancement within the fundus of the right internal auditory canal, suggestive of infectious, post-infectious, or inflammatory neuritis of the right facial nerve, with no evidence of acute infarct or hemorrhage.

**Figure 2:** MRI of the head showing focal enhancement in the lateral right internal auditory canal (arrows). (A) T1-weighted coronal view. (B) T1-weighted axial view

The patient was treated with an eye patch, carboxymethylcellulose eye drops, and a 10-day course of oral prednisone. He was discharged to inpatient rehabilitation and later transitioned home with continued physical therapy. At two-week follow-up, right facial paralysis had improved, though diplopia persisted.

All information in this case report is de-identified. Informed consent was obtained from the patient for publication.

## Discussion

GBS comprises a spectrum of acute demyelinating motor and sensory polyneuropathies most often triggered by infection and, less commonly, immunization. The estimated global incidence is about 1.8 per 100,000 per year between 1980 and 2008, with risk increasing with age [4]. First described in 1916, GBS is characterized by diminished or absent deep tendon reflexes and albuminocytological dissociation in cerebrospinal fluid [5]. The most common subtype, acute inflammatory demyelinating polyradiculoneuropathy (AIDP), primarily affects the limbs and presents with symmetric ascending paralysis and numbness. Cervical and bulbar involvement may occur, and disease progression can rapidly impair respiratory function. Autonomic dysfunction is also possible, leading to hemodynamic instability, ileus, or urinary incontinence. Although GBS is a clinical diagnosis, CSF analysis often supports it by showing elevated protein without pleocytosis, as in our patient. Electromyography, when performed, may demonstrate findings consistent with a demyelinating process.

This case describes a 65-year-old man with a preceding URI who presented with two days of progressive lower extremity weakness and later developed unilateral facial droop eight days into his course. Cranial nerve palsies occur in about half of GBS cases, but they are usually bilateral and appear early, alongside limb weakness. The facial nerve is most often affected, leading to facial diplegia, though extraocular, pharyngeal, lingual, and cervical muscles may also be involved. Reports of unilateral facial palsy are rare, and even fewer describe onset after partial recovery of limb strength [6]. In a 2021 review, Huang et al. identified 28 cases of delayed-onset facial paralysis across seven studies, with 13 (46.4%) being unilateral and most showing involvement of additional cranial nerves, particularly ophthalmoplegia [6]. Because our patient’s cranial nerve impairment developed two days after completing IVIG, treatment-related fluctuation (TRF) was considered. TRFs occur in 8%-6% of GBS patients and are defined as new or worsening neurological deficits after initial improvement or stabilization following IVIG or plasmapheresis. Diagnostic criteria require a ≥5 point decline in Medical Research Council (MRC) sum score or ≥1 grade worsening in Hughes disability score within weeks of treatment [7]. Since these metrics heavily weight limb weakness and facial hemiplegia does not significantly lower functional scores, our patient did not meet current TRF definitions. Moreover, he lacked known TRF risk factors such as cytomegalovirus infection, delayed nadir, or comorbidities. Thus, while his case highlights a limitation of existing TRF criteria, it more likely represents a rare subset of GBS patients with delayed-onset unilateral facial palsy, reflecting either atypical disease progression or insufficient response to therapy.

Another notable feature in our patient was the unilateral facial nerve hyperintensity seen on gadolinium-enhanced MRI. While cauda equina root enhancement is occasionally observed on lumbosacral MRI, brain imaging in GBS is usually normal, even in cases with cranial nerve palsies. One of the earliest reports was of a 27-year-old woman with distal extremity weakness and facial diplegia, in whom bilateral facial nerve enhancement was detected [8]. Fulbright et al. later described a 50-year-old woman with unilateral lower limb weakness that progressed to dysphagia and bilateral facial weakness, where MRI revealed enhancement of bilateral cranial nerves VI and the right cranial nerves VII, X, and XI [9]. Interestingly, electrodiagnostic studies showed demyelination of the left facial nerve, which was not enhanced, and the abducens nerve enhancement had no clinical correlate of ophthalmoplegia [9]. Such inconsistencies may reflect the heterogeneity of GBS pathophysiology. The same immune-mediated process believed to underlie limb weakness is generally assumed to extend to cranial nerves, with both cellular and humoral mechanisms implicated [1]. Some authors, particularly in pediatric cases, have proposed that facial palsy may also result from compression within the facial canal due to edema and hemorrhage secondary to GBS-related hypertension [10]. In reports of cauda equina enhancement, radiologic resolution has paralleled clinical recovery, but there is not yet enough evidence to draw the same conclusion for cranial nerve involvement. We encourage clinicians, when feasible, to identify potential infectious triggers and obtain both MRI and serologic studies, as these may provide insight into the variable manifestations of GBS.

Though GBS is generally self-limiting, with peak disability reached around four weeks, timely administration of plasma exchange (PE) or intravenous immunoglobulin (IVIG), as in our case, can shorten recovery. Severe cases may require ICU monitoring for rapid intervention in the event of cardiopulmonary complications [1]. Facial hemiplegia associated with GBS may precede or follow limb weakness and can be mistaken for Bell’s palsy, underscoring the importance of distinguishing it from atypical GBS variants to guide management. Corticosteroids, the standard therapy for Bell’s palsy, were started empirically in our patient due to diagnostic uncertainty, but they are not recommended in GBS, as studies have shown limited benefit and potential harm [1]. To date, no systematic studies address the treatment of GBS with delayed-onset facial palsy. Standard therapies such as IVIG and PE remain the mainstay, though prior reports suggest that most cases resolve within about three weeks regardless of treatment [6].

## Conclusions

GBS is a heterogeneous condition with diverse clinical presentations. Awareness of its rare variants is essential, as they may mimic other disorders and delay diagnosis, increasing the risk of morbidity and mortality. The focal gadolinium enhancement of cranial nerves observed in our patient suggests that blood-brain barrier impairment may contribute to this GBS phenotype. We encourage clinicians to pursue a comprehensive evaluation in atypical cases, including MRI, electrophysiology, serology, and infectious workup, to better characterize these variants and identify associated features.
